# Spatial Pattern Evaluation of Rural Tourism via the Multifactor-Weighted Neural Network Model in the Big Data Era

This article has been retracted.

**DOI:** 10.1155/2021/5845545

**Published:** 2021-08-27

**Authors:** Jiangrui Zhu, Feng Jian

**Affiliations:** School of Culture and Tourism, Ningxia University, Zhongwei 755000, China

## Abstract

The exploration of the evaluation effect of rural tourism spatial pattern based on the multifactor-weighted neural network model in the era of big data aims to optimize the spatial layout of rural tourist attractions. There are plenty of problems such as improper site selection, layout dispersion, and market competition disorder of rural tourism caused by insufficient consideration of planning and tourist market. Hence, the multifactor model after simple weighting is combined with the neural network to construct a spatiotemporal convolution neural network model based on multifactor weighting here to solve these problems. Moreover, the simulation experiment is conducted on the spatial pattern of rural tourism in the Ningxia Hui Autonomous Region to verify the evaluation performance of the constructed model. The results show that the prediction accuracy of the model is 97.69%, which is at least 2.13% higher than that of the deep learning algorithm used by other scholars. Through the evaluation and analysis of the spatial pattern of rural tourist attractions, the spatial distribution of scenic spots in Ningxia has strong stability from 2009 to 2019. Meanwhile, the number of scenic spots in the seven plates has increased and the time cost of scenic spot accessibility has changed significantly. Besides, the change rate of the one-hour isochronous cycle reaches 41.67%. This indicates that the neural network model has high prediction accuracy in evaluating the spatial pattern of rural tourist attractions, which can provide experimental reference for the digital development of the spatial pattern of rural tourism.

## 1. Introduction

Nowadays, with the close integration between information technology and the tourism industry, the Internet, big data, and artificial intelligence have rapidly become the hot technologies of industrial development. Especially, relevant incentive policies issued by the government and increased financial subsidies, which encourage the development of tourism and other projects in remote mountain villages, have injected new vitality into rural development and brought significant economic growth. However, some problems have appeared in rural tourism, such as improper site selection, layout dispersion, construction repetition and inefficiency, and market competition disorder, during the accelerated development as a result of improvident consideration of the planning basis and tourist market [1, 2]. Therefore, the application of artificial intelligence and big data analysis technology to the optimization of the spatial structure of rural tourism has become the focus of scholars in the current relevant fields.

The tour is a kind of sightseeing and entertainment activity on the premise of the coexistence of human society and natural environment. In recent years, the advocacy of “lucid waters and lush mountains are invaluable assets” and related documents on rural tourism have been proposed by the Chinese central government, which has become an important guiding force for the efficient and rapid development of rural tourism in China [3]. The Ningxia Hui Autonomous Region is one of the minority concentrated areas in northwest China. It puts ecological environment protection in the first place under the “The Belt and Road Initiative” policy and the economic protection strategy in the Yellow River Basin. Meanwhile, Ningxia is working hard to ensure ecological security in the middle and upper reaches of the Yellow River and achieve the goal of building a beautiful China. Furthermore, due to the topography in Ningxia, more than 80% of the tourism resources are concentrated in rural areas, which have become the largest potential area for tourism development in the province with obvious advantages over the whole country [4]. The unique natural resources and geographical environment and other ecological advantages in Ningxia promote rural tourism into an important force progressing fast in the economic development of Ningxia. Meanwhile, a series of relevant policies issued by the government not only provide strong support for the development of rural tourism but also clarify the specific development direction and planning. This makes the number of rural tourism spots in Ningxia show rapid growth momentum in recent years.

With the rapid increase in rural tourist attractions, changes in economy, policy, and traffic changes have a deepening impact on rural tourism, resulting in the transformation of the spatial pattern of rural tourism. The rapid development in rural tourism also increases the demand for corresponding tourism space, which intensifies the contradiction between supply and demand of space in the region and leads to the imbalance of spatial utilization structure in the region [5]. In other words, the fast development of the economy and living standards of the people has also destroyed the original, pure, and natural environment artificially. In recent years, artificial intelligence technologies, such as big data analysis and artificial neural networks, have been widely used in various industries, such as machine translation, image recognition, and natural language processing. Deep learning, as one of the artificial intelligence algorithms, can learn multilevel features of data from raw data such as the spatial pattern of the original geographical environment without the participation of experts in related fields, which greatly saves the cost of labor, material and time [6, 7]. Meanwhile, the deep learning algorithm can classify tasks according to the important characteristics learned, which has far-reaching engineering practice value in the spatial pattern evaluation of rural tourism.

In summary, the evaluation and analysis of the spatial pattern of rural tourism are of great practical value for the development of tourism. The innovations of the existing research are as follows:

- Taking Ningxia Hui Autonomous Region in Northwest China as the research object, the research evaluates the spatial pattern of rural tourism.
- The research analyzes the confusion of rural tourism location and scattered layout caused by insufficient consideration of various factors such as the planning basis of rural tourism.
- Based on the simple weighting of the multifactor model, combined with neural network, the research constructs a spatiotemporal convolution neural network model based on multifactor weighting. Finally, the evaluation effect of rural tourism spatial pattern is analyzed through simulation.

The research is structured as follows: Section 1 is the introduction that mainly explains the current situation and background of rural tourism and the research purpose and significance.  Section 2 is the related works, which mainly analyzes the research status of scholars related to rural tourism and algorithms.  Section 3 mainly constructs and evaluates the model of rural tourism spatial pattern based on multifactor-weighted neural network algorithm.  Section 4 is the results and discussion. After the simulation of the rural tourism spatial pattern model, its performance is analyzed and discussed more clearly.  Section 5 is the conclusion that summarizes the research methods and results to provide basis for follow-up research.  Section 6 is future work, which analyzes the shortcomings, and explains the follow-up research.

## 2. Related Works

### 2.1. Current Situation of Rural Tourism Development

At present, with the accelerating process of urbanization and the rapid improvement of people's living standards, people pay more attention to their spiritual needs while satisfying material needs. As one of the rural revitalization strategies advocated by the state, rural tourism has been studied by many scientific researchers. Su et al. [8] adopted a mixed methods research design, including quantitative questionnaires and qualitative semistructured interviews, to analyze tourism and rural sustenance at Hetu Town, Anhui Province, China. They found that the utilization of synergistic relationships between tourism and other sources of income could improve the overall livelihood sustainability. Meanwhile, they discussed the practical significance to enhance tourism participation and ensure appropriate benefit sharing with an emphasis on the roles of government [8]. Guaita Martínez et al. [9] demonstrated that tourism was a key sector in the sustainable development of rural environments. Hence, they proposed a more comprehensive and objective method to compare the level of seasonality of a group of rural destinations with that of coastal and urban destinations. Through the study, they found that the methodology enabled them to identify, which variables explained the differences in the level of seasonality of each destination to a large extent. Finally, the research results showed that the variables that do so are related to the internalization of the destination and changes in the availability of bed places [9]. Cunha et al. [10] explored the motivation, management practices, and consequences of rural tourism entrepreneurs considering data obtained from eight small tourism accommodation units, whose owners participated in semistructured interviews. The results revealed long-term planning and tend to form robust networks of entrepreneurs, which clearly contributed to not only the establishment of a dynamic but also more sustainable entrepreneurial ecosystem of tourism in rural areas [10]. Chi and Han [11] took Anji County as a case to comprehend the role of rural tourism destination performances in affecting destination image and predicting satisfaction and loyalty and verified the moderating effect of tourists' expectation [11]. These above works can provide certain guidance and reference for scholars and rural tourism practitioners to deepen the research on tourism expectations, rural tourism performance, destination image, and the relationship between tourist satisfaction and loyalty.

### 2.2. Application Status of Neural Network Algorithms in Tourism

Today, neural networks are widely used in diverse industries, and many researchers have analyzed its application in emerging tourism. Lee et al. [12] analyzed the prediction performance of backpropagation neural networks (BPNNs), radial basis function networks (RBFNs), probabilistic neural networks (PNNs), and clustered probabilistic neural networks (CPNNs) in tourism. They found that PNNs performed best in all artificial neural networks, especially showing extreme accuracy in predicting underrepresented modes [12]. Petersen et al. [13] proposed a system for bus travel time prediction that leveraged the nonstatic spatiotemporal correlations present in urban bus networks, allowing the discovery of complex patterns not captured by traditional methods. Finally, they found that the multioutput, multitime step, deep neural network using a combination of convolutional and long short-term memory (LSTM) significantly outperformed all the other comparative methods [13]. Abdollahi et al. [14] proposed a multistep deep learning-based algorithm for predicting travel time. They found that feature extraction and clustering algorithms could be used to improve the feature space, which was robust [14]. Hu et al. [15] used artificial neural network (ANN) simulation to reveal the characteristics of human activity patterns and urban functions. They demonstrated that the proposed method, with relatively less loss and high accuracy, outperformed other comparative methods for classifying urban functions at the road segment level. Besides, they believed that their work contributed to the assessment of urban functional structure and further aid urban planners in designing better urbanization strategies with regard to traffic interaction and urban space structure [15].

Through the above scholars' research, most of the current research on rural tourism focuses on tourism resources, tourism development, tourism development mode, problems, and countermeasures, etc., while focusing little on the spatial structure of rural tourism and the spatial problems. Moreover, the application of applying deep learning to tourism is mainly in the prediction of travel time rather than in the design of tourism spatial pattern. Therefore, the neural network is introduced into the simply weighted multifactor model to construct a multifactor-weighted neural network model to evaluate the spatial pattern of rural tourism with the research object of rural tourist attractions in Ningxia.

## 3. Construction and Evaluation of Rural Tourism Spatial Pattern Based on Multifactor-Weighted Neural Network Algorithm

### 3.1. Overview of the Study Area

Ningxia Hui Autonomous Region is referred to as Ningxia, and Yinchuan is its provincial capital. Located in the northwest inland area of China, east of Shaanxi, west and north of Inner Mongolia, and south of Gansu, Ningxia occupies a total area of 66,400 square kilometers, located in the northwest of the four geographical divisions [16]. The terrain in Ningxia gradually tilts from southwest to northeast, with hills and ravines standing in numbers, consisting of three plates: the northern Yellow River irrigation area, the central arid zone, and the southern mountainous area. The autonomous region is located in the Yellow River water system, and the terrain is high in the south and low in the north, showing a ladder-like decline. The whole region is located in the continental arid and semiarid climate zone [17]. Ningxia Hui Autonomous Region administrates 5 prefecture-level cities (9 municipal districts, 2 county-level cities, and 11 counties), with two national AAAAA-level tourist attractions of the China Western Film Studio in Zhenbeibu and the Sand Lake, several 4A-level tourist attractions (including 96 A-level scenic spots), and numerous rural scenic spots [18]. There are mainly seven tourism plates in Ningxia: Great Sand Lake Holiday and Leisure Area, Xixia Cultural Tourism District, Saishang Hui Township Cultural Experience Plate, Frontier Cultural Tourism Plate, Great Shapotou Resort and Leisure Plate, Weizhou Historical and Cultural Tourism Plate, and Great Liupan Red Ecological Resort Plate [19]. Among them, the study area in Ningxia is shown in Figure 1.

### 3.2. Analysis on the Goal of Rural Tourism Pattern Construction

The spatial pattern of rural tourism not only affects the spread and flow of people, materials, and information in rural tourism activities but also guarantees the normal and orderly operation of various functions of rural tourism. Under the rapid development of the social economy, people's diversified spiritual needs have brought good opportunities for the development of rural tourism. However, mature rural tourism has cumulatively higher requirements for spatial patterns, which have an increasingly obvious impact on rural tourism. The requirements of rural tourism on the spatial pattern are mainly reflected in the rational utilization of resources, the correct guidance of the market, and the reasonable layout of products, as shown in Figure 2.

As shown in Figure 2, firstly, the rational development and utilization of rural tourism resources play an important role in the long-term and orderly development of rural tourism activities. Moreover, the construction of the spatial pattern can ensure the rational use of rural tourism resources and the maximum utilization of the developed parts. Secondly, the correct guidance of the rural tourism market requires the spatial pattern to ensure the accurate implementation of rural tourism market positioning and planning. Thirdly, the spatial pattern of multilayer structure can meet the multilayer structure of tourism products and ensure the priority of core products in rural tourism activities. Besides, the spatial pattern and multilevel system of tourism products can better meet the diversified needs of different tourists [20]. Similarly, the spatial pattern of rural tourism can affect the function and structure of rural tourism, which makes rural tourism a multifunctional leisure activity with different functions from different perspectives. Meanwhile, the integrity of tourists' rural experience is guaranteed.

The spatial structure of rural tourism is the organization rules of functional zoning, tourism resources pattern, and tourism product pattern, to ensure the orderly conduct of tourism activities. The construction of rural tourism spatial pattern is not only the planning and organization of rural tourism function and structure but also the dissection and integration of the spatial base. The construction of the spatial pattern here lies in the following three objectives: first, to ensure good development of rural tourism; second, to utilize and protect resources reasonably; and third, to allocate rural tourism products properly.

### 3.3. Construction and Analysis of the Multifactor-Weighted Neural Network Algorithm Model

It is necessary to select suitable factors and models to construct the multifactor model. If the process of building a multifactor model is likened to the production process of the factory, the factor will be the raw material, and the model will be the production line. With given raw materials, the choice of different production lines means different processing technology and different results correspondingly. Usually, the construction of multifactor model can be divided into the simple additive weight, linear regression method, and artificial intelligence approach. Although the simple additive weight can calculate the weighted average of each factor, it is impossible to predict the internal factors. Therefore, the multifactor model under simple additive weight is combined with neural network to construct a multifactor-weighted neural network model to evaluate the spatial pattern of rural tourism.

As the core algorithm of the model, neural network algorithm is very important to understand the role of data sources related to the spatial pattern of rural tourism. In the neural network algorithm system, CNN is the fastest growing feedforward neural network model with the best performance with the biggest advantage of local connection and weight sharing. Numerous neurons in CNN are organized in a certain way to respond to the overlapping areas in the vision field [21]. In CNNs, the first parameter of its operation is called the input and the second parameter (function *w*) is called the kernel function. The output is sometimes called the feature map [22]. Usually, CNNs perform convolution operations on multiple dimensions. Substitute a two-dimensional matrix *I* into the input and a two-dimensional kernel *K*, then the following equation is obtained:

(1) $$\begin{array}{c} S\left(i,j\right)=\left(I\cdot K\right)\left(i,j\right)=\sum_{m}\sum_{n}I\left(m,n\right)K\left(i-m,j-n\right), \end{array}$$

where *i*, *j*, *m*, and *n* are fixed parameters, representing the dimension and order of the matrix. The exchange of convolutions can be equivalently written as

(2) $$\begin{array}{c} S\left(i,j\right)=\left(I\cdot K\right)\left(i,j\right)=\sum_{m}\sum_{n}I\left(i-m,j-n\right)K\left(m,n\right). \end{array}$$

The exchangeability feature of convolution operation is caused by the kernel flip corresponding to the input. The index of kernel is decreasing with the increase of the index of input. The only purpose of kernel flip is to achieve exchangeability. Although exchangeability is useful in proving, it is not an important property in the application of neural networks. In contrast, many neural networks have a correlation function called cross-correlation function [23], which is almost identical to the convolution operation but cannot flip the kernel, as presented in

(3) $$\begin{array}{c} S\left(i,j\right)=\left(I\cdot K\right)\left(i,j\right)=\sum_{m}\sum_{n}I\left(i+m,j+n\right)K\left(m,n\right). \end{array}$$

Any neural network algorithm that uses matrix multiplication but does not depend on the special properties of matrix structure is suitable for convolution operation without great modification. The working principle of CNN is to update the control weight *w* and bias *b* by continuously adjusting the learning rate *γ* and minimize the loss function, so as to obtain the predicted value closest to the real value [24]. Typical CNNs usually use three important ideas, namely, sparse interaction, parameter sharing, and equivariant representation, to improve the machine learning system, in order to deal with large-scale input more effectively.

The spatiotemporal graph convolution network (STGCN) is proposed after combining the spatial pattern and time characteristics of rural tourism. The spatial characteristics of rural structure can be extracted by graph convolution. In the time dimension, the one-dimensional convolution and the gating linear unit are used to extract the short-term evolution dependence of the spatial pattern. The two are alternately fused to form a spatiotemporal convolution block. Finally, the model structure is built on a stack of spatiotemporal convolution blocks. The feature extraction of rural tourism spatial pattern based on multifactor-weighted spatiotemporal CNN algorithm is illustrated in Figure 3.

The network structure of rural tourism spatial pattern is a general topological graph, where the weight of each factor may not be equal. Therefore, the two-dimensional convolution commonly used in CNNs is not applicable in the topological graph but more suitable for Euclidean structures with grid data. Here, similar convolution operations need to be defined in general graphs to extract spatial features. The graph convolution operator “∗*G*” is introduced based on the definition of spectral graph convolution, that is, the transformation of the signal *x* ∈ *R*^*n*^ by a kernel Θ, as shown in

(4) $$\begin{array}{c} \Theta_{*G}x=\Theta \left(L\right)x=\Theta \left(U\wedge U^{T}\right)x=U\Theta \left(\wedge \right)U^{T}x. \end{array}$$

In equation (4), *L* refers to the normalized Laplacian matrix *L*=*I*_*n*_ − *D*^−1/2^*WD*^1/2^ of the network graph for the spatial pattern, where *I*_*n*_ denotes the *n*-order unit matrix, *D* ∈ *R*^*n*×*n*^ is the degree matrix of the network graph, *D*_*ii*_=∑_*j*_*w*_*ij*_, and *W* ∈ *R*^*n*×*n*^ represents the weight matrix of the network graph. Besides, *U* ∈ *R*^*n*×*n*^ is the Fourier basis, which is the matrix composed of the eigenvectors of *L*, that is, *L*=*U*∧*U*^*T*^. Finally, ∧∈*R*^*n*×*n*^ means the matrix is composed of the eigenvalues of *L*.

In the actual calculation, Chebyshev polynomials can be used to avoid matrix feature decomposition and reduce computational complexity. In the Chebyshev polynomials of *K* − 1-order, the approximate kernel is Θ. *K* is the size of the convolution kernel (Kernel size) of the graph, similar to the size of the traditional convolution operation, which determines the maximum radius of the convolution starting from the center node [25]. Thus, graph convolution can be written as follows:

(5) $$\begin{array}{c} \Theta_{*G}x=\Theta \left(L\right)x\approx \sum_{k=0}^{K-1}\theta_{k}T_{k}\left(\tilde{L}\right)x, \end{array}$$

where $\tilde{L}$ represents a scaled Laplacian matrix $\tilde{L}=\left(2L/\lambda_{\max}\right)-I_{n}$ and *θ*_*k*_ is a network parameter to be learned. *T*_*k*_ signifies a *k*-order Chebyshev polynomial determined by the following recursive relation expressions:

(6) $$\begin{array}{c} T_{0}\left(x\right)=1,\\ T_{1}\left(x\right)=x,\\ T_{n+1}\left(x\right)=2xT_{n}\left(x\right)-T_{n-1}\left(x\right). \end{array}$$

The complexity of graph convolution calculation can be reduced from *O*(*n*^2^) to *O*(*K*|*ε*|) through *K* approximation cores Θ of the Chebyshev polynomial.

Using the same convolution kernel Θ in *M* time steps in the rural tourism spatial pattern, the graph convolution can be used on the three-dimensional tensor of the rural tourism spatial pattern. The output of a single convolution kernel at each time step is an *n*-dimensional vector *R*^*n*^. The output of *C*_*o*_ (*o* means output or the number of channels for the output vector, i.e., the extraction of features of different factors in the spatial pattern network) convolution kernels at each time step is *R*^*n*×*C*_*o*_^, and the output at all time steps is *R*^*M*×*n*×*C*_*o*_^.

Then, the feature of rural spatial pattern is extracted by the STGCN. The input of the time convolution of each vertex can be regarded as a sequence of length *M*, with *Ci* channels (*i* denotes the input or the number of channels of the input vector), written as *Y* ∈ *R*^*M*×*C*_*i*_^. Besides, the convolution kernel is Γ ∈ *R*^*K*_*t*_×2*C*_0_×*C*_*i*_^, and *Y* is mapped to the result. Time-gated convolution can be defined as follows:

(7) $$\begin{array}{c} \Gamma_{*T}Y=P⊗\sigma \left(Q\right)\in R^{\left(M-K_{t}-1\right)\times C_{o}},\\ P=W_{1}Y+b_{1}\in R^{\left(M-K_{t}-1\right)\times C_{o}},\\ Q=W_{2}Y+b_{2}\in R^{\left(M-K_{t}-1\right)\times C_{o}}, \end{array}$$

where *P* and *Q*, respectively, refer to the input gates of GLU (gated linear unit), and each of them uses different *C*_*o*_ (*o* means output or the number of channels for the output vector, i.e., the extraction of features of different factors in the spatial pattern network) convolution kernel parameters to perform linear transformation on the input vector *Y*. Furthermore, *W*_*i*_ and *b*_*i*_ are the corresponding weight and bias parameter. ⊗ refers to the Hadamard product. *σ* represents the sigmoid activation function commonly used in neural networks, and the nonlinear gate *σ* (*Q*) controls the information entering the model in *P*. Compared with the activation function value directly using linear transformation, the structure can better excavate the complex time characteristics of rural spatial pattern [26]. The input and output of spatiotemporal convolution blocks are three-dimensional tensors. The input of the *l*-th spatiotemporal convolution block is *v*^*l*^ ∈ *R*^*M*×*n*×*C*^*l*^^, and its output is *v*^*l*+1^ ∈ *R*^(*M* − 2(*K*_*t*_ − 1))×*n*×*C*^*l*+1^^, which is gained by

(8) $$\begin{array}{c} v^{l+1}=\Gamma_{2*T}^{l}\text{RELU}\left(\Theta_{*G}^{l}\left(\Gamma_{1*T}^{l}v^{l}\right)\right). \end{array}$$

Here, Γ_1*∗T*_^*l*^ and Γ_2*∗T*_^*l*^ are the upper time convolution and lower time convolution in the *l*-th spatiotemporal convolution block. Moreover, Θ_*∗G*_^*l*^ is the graph convolution in the middle, and RELU stands for the activation function of the linear correction unit.

Data are mapped to the predicted flow to further extract the temporal and spatial characteristics in the rural spatial pattern. Meanwhile, the output of the last spatiotemporal convolution block is introduced into the output layer composed of two temporal convolutions and a fully connected layer. The output result of the output layer is the predicted value of the next step, combined with the original data to reconstruct $x=\left(x_{2},\ldots ,x_{t},{\hat{x}}_{t+1}\right)$. Then, the predicted value of the next step is obtained through the model until obtaining the predicted value of the future *H*-th step [27]. The optimization loss function of the whole model can be written as

(9) $$\begin{array}{c} L\left(\hat{v};W_{\theta }\right)=\sum_{t}{\left\|\hat{v}\left(v_{t-M+1},\ldots ,v_{t},W_{\theta }\right)-v_{t+1}\right\|}^{2}. \end{array}$$

In equation (9), *W*_*θ*_ refers to the weight training parameters in the model, *v*_*t*+1_ denotes the real value of the future, and $\hat{v}\left(\cdot \right)$ shows the prediction of the model.

According to the convolution operation *σ*(*Wx*+*b*) in CNNs, the graph convolution operation can be defined as *σ*(Θ*Lx*) below, where *W* and *b* in the former and Θ in the latter are the parameters to be learned, as follows:

(10) $$\begin{array}{c} \Theta_{*G}x=\sigma \left(g_{\theta }\left(L\right)x\right)=\sigma \left(g_{\theta }\left(U\wedge U^{T}\right)x\right)=\sigma \left(Ug_{\theta }\left(\wedge \right)U^{T}x\right),\\ g_{\theta }\left(\wedge \right)=\left(\begin{array}{c} \theta_{1}\\ \ddots \\ \theta_{n} \end{array}\right). \end{array}$$

To avoid matrix eigenvalue decomposition and reduce the number of parameters, *g*_*θ*_(∧) can be improved as

(11) $$\begin{array}{c} g_{\theta }\left(\wedge \right)=\left(\begin{array}{c} \sum_{j=0}^{K}\alpha_{j}\lambda_{1}^{j}\\ \ddots \\ \sum_{j=0}^{K}\alpha_{j}\lambda_{n}^{j} \end{array}\right). \end{array}$$

Thus, equation (12) can be obtained as

(12) $$\begin{array}{c} \Theta_{*G}x=\sigma \left(Ug_{\theta }\left(\wedge \right)U^{T}x\right)=\sigma \left(\sum_{j=0}^{K}\alpha_{j}L^{j}x\right). \end{array}$$

To avoid computing matrix multipliers, it is proved that equation (12) can be approximated by *k* − 1–order Chebyshev polynomial, as shown in

(13) $$\begin{array}{c} \Theta_{*G}x=\sigma \left(L\right)x\approx \sum_{k=0}^{K-1}\theta_{k}T_{k}\left(\tilde{L}\right)x. \end{array}$$

Among them, *θ*_*k*_ is the network parameters to be learned. Equation (13) is used as the graph convolution operation of the first layer to integrate the information of *k* nodes around the node. Thus, the spatial pattern characteristics of multiple channels can be obtained through several groups of different parameters *θ*_*k*_.

The square error is used as the loss function here, and the optimization objective can be expressed as

(14) $$\begin{array}{c} \underset{\Theta }{\min}\sum_{t\in \text{Train}}{\left\|y_{t}-{\overset{⌢}{y}}_{t}\right\|}_{F}^{2}, \end{array}$$

where Θ is the parameters to be learned in the graph convolution layer, whereas *y*_*t*_ is the real flow at time *t* and ${\overset{⌢}{y}}_{t}$ is the predicted flow. Meanwhile, the objective function is optimized by the Adam optimization algorithm to conduct the subsequent calculation and parameter solution.

The training of the proposed model mainly includes the learning rate updating strategy through the “Poly” learning rate adjustment method via the polynomial attenuation [28], as shown in

(15) $$\begin{array}{c} \text{init}\_\text{lr}\times {\left(1-\frac{\text{epoch}}{\max\_\text{epoch}}\right)}^{\text{power}}. \end{array}$$

In equation (15), the initial learning rate init_lr is 0.0005 (5*e*^−4^) and the power is set as 0.9.

### 3.4. Data Sources of the Spatial Pattern of Rural Tourism in the Study Area

The research data of rural tourist attractions are from the list of rural tourist attractions published by the official website of the Department of Culture and Tourism of Ningxia Hui Autonomous Region (http://whhlyt.nx.gov.cn/) in 2009 and 2019. Besides, the basic road data comes from the 1 : 10,000,000 national basic geographic database released by the National Dynamic Atlas (http://www.webmap.Cn). Finally, the administrative boundary data of the villages come from the standard map service website of the Department of Natural Resources of Ningxia Hui Autonomous Region (http://zrzyt.nx.gov.cn/).

### 3.5. Simulation Analysis

The MATLAB network simulation software is used for the simulation analysis of the performance of the multifactor-weighted spatiotemporal CNN algorithm. The data resource has been explained in the previous section. The obtained data are divided into the training set, verification set, and test set according to the proportion of 60%, 20%, and 20%, respectively.

The hyperparameters of the constructed neural network model are set as the following: the number of iterations is 60, the simulation time is 2000 s, and the batch size is 128. In the performance analysis of the proposed model, the prediction performance is compared with other algorithms applied by other scholars in related fields from the perspectives of accuracy, precision, recall, and *F*1 values (weighted harmonic mean of precision and recall). The comparative algorithms include LSTM [29], Bi-directional long short-term memory (BiLSTM) [30], the AlexNet improved by Visual Geometry Group (VGGNet) [31], AlexNet [32], and STGCN [33]. Furthermore, both hardware and software configurations are considered in the specific simulation experiment. The software is equipped with the Linux 64-bit operating system and Python 3.6.1, along with the PyCharm development platform. The CPU of the hardware is Intel core i7-7700 @ 4.2 GHz of 8 core, with the memory of Kingston ddr4 2400 MHz of 16G, and the GPU is Nvidia GeForce 1060 of 8G.

The following indicators are mainly taken into account in the use of the obtained data to evaluate the spatial pattern of rural tourism. Firstly, the nearest neighbor distance index (NNI). The calculation result of the average distance between the closet attractions is compared with that between nodes in the random distribution to analyze the degree of deviation from the random distribution, so as to obtain the distribution type of rural tourism attractions [34]. The calculation can be written as

(16) $$\begin{array}{c} \text{NNI}=\frac{\left[\sum_{i=1}^{N}\min\left(d_{ij}\right)/N\right]}{\sqrt[{0.5}]{A/N}}w_{i}. \end{array}$$

In equation (16), min (*d*_*ij*_) refers to the distance between any scenic spot *i* and its nearest scenic spot *j*; *N* is the total number of rural scenic spots; and *A* is the total area of the study area. NNI ≤ 0.5 is generally considered as aggregate, with 0.5 < NNI ≤ 0.8 as aggregate random, 0.8 < NNI ≤ 1.2 as random, 1.2 < NNI ≤ 1.5 as random discrete, and NNI > 1.5 as uniform.

Secondly, the standard deviation ellipse mainly reflects the moving direction of the centroid of the scenic spot space. Suppose a region has *n* subregions, (*x*_*i*_, *y*_*i*_) is the center coordinates of the *i*-th region and *w*_*i*_ is the attribute value and weight of the *i*-th subregion [35]. The standard deviation ellipse can be expressed as

(17) $$\begin{array}{c} M\left(\bar{X},\bar{Y}\right)=\left[\frac{\sum_{i=1}^{n}w_{i}x_{i}}{\sum_{i=1}^{n}w_{i}}\times \frac{\sum_{i=1}^{n}w_{i}y_{i}}{\sum_{i=1}^{n}w_{i}}\right]. \end{array}$$

Third, the time cost of accessibility of the scenic spot. The accessibility is quantitatively analyzed by the minimum time spent by tourists, and the small value demonstrates the good accessibility [36], which can be expressed as

(18) $$\begin{array}{c} T_{i}=\text{Exp}\left(i,j\right). \end{array}$$

In equation (18), *T*_*i*_ represents the accessibility of site location *i* of the scenic spot *j*, whereas Exp (*i*, *j*) denotes the minimum time-consuming function to calculate the traffic between *i* and *j*. Among them, the isochronous circle is mainly divided into six parts: <1 h, 1-2 h, 2-3 h, 3-4 h, 4-5 h, and >5 h.

## 4. Results and Discussion

### 4.1. Comparative Analysis of Prediction Performance of Each Model Algorithm

The comparative analysis is conducted on the spatiotemporal convolution neural network algorithm based on multifactor weighting to study the prediction performance of the constructed model on the spatial pattern of rural tourism. The constructed model is compared with LSTM, BiLSTM, VGGNet, AlexNet, and STGCN from the perspective of accuracy, precision, recall, and *F*1 values, with the results shown from Figures 4to 7.

According to the results presented from Figures 4to 7, the accuracy of the constructed model reaches 97.69%, which is at least 2.13% higher than that of the deep learning algorithms (including LSTM, BiLSTM, VGGNet, AlexNet, and STGCN) used by other scholars. Besides, the neural network model has the highest precision, recall, and *F*1 value, and the *F*1 value may be smaller than the precision and recall rather than be between them. Therefore, compared with the deep learning algorithm adopted by other scholars, the spatiotemporal CNN algorithm based on multifactor weighting has better prediction accuracy and better performance in evaluating the spatial pattern of rural tourism.

### 4.2. Spatial Pattern Evaluation of Rural Tourist Attractions

In the spatial pattern evaluation of rural tourist attractions, the spatial pattern of rural tourist attractions in the seven tourism plates of Ningxia Hui Autonomous Region in 2019 is compared with that in 2009. The spatial distribution concentration, spatial centroid mobility, and spatial connection accessibility of rural tourist attractions are expatiated from Figures 8to 10.

The NNI of the seven tourism plates is shown in Figure 8. It can be found that the spatial distribution concentration of rural attractions in Ningxia Hui Autonomous Region does not change significantly at the provincial level. The NNI in 2009 was 0.57, and the spatial structure type was aggregate-random. The NNI in 2019 was 0.69 increasing by 0.12. Meanwhile, the random distribution trend of attractions increases, but the spatial structure type was still aggregate-random, showing strong stability. The concentration of spatial distribution of scenic spots was analyzed from various tourism plates. Among them, the NNI of the Great Sand Lake Holiday and Leisure Area in 2009 was 0.67, with the aggregate-random distribution type, compared with the NNI of 0.48 and the aggregate distribution type in 2019. In 2009, the NNI of the Xixia Cultural Tourism District was 0.62 with the aggregate-random distribution type, compared with the NNI of 0.45. Besides, the agglomeration trend of scenic spots increased and the spatial structure type changed from aggregate-random to aggregate. In 2009, the NNI of the Saishang Hui Township Cultural Experience was 1.12 with the random distribution type of scenic spots, compared with the NNI of 0.63 in 2019. Meanwhile, the agglomeration trend of scenic spots increased, changing into the aggregate-random distribution type. In 2009, the NNI of the Frontier Cultural Tourism Plate was 0.75 with the aggregate-random distribution type of scenic spots, compared with the NNI of 0.56 in 2019. The agglomeration trend of scenic spot distribution also increased, but the spatial structure type did not change. In 2009, the NNI of the Great Shapotou Resort and Leisure Plate was 0.86 with the random distribution type of scenic spots, compared with the NNI of 0.61 in 2019. Furthermore, the agglomeration trend of scenic spot distribution increased, and the spatial structure type changed from aggregate-random to aggregate-random. In 2009, the NNI of the Weizhou Historical and Cultural Tourism Plate was 0.94 with the random distribution type of scenic spots, compared with the NNI of 0.48 in 2019. Besides, the agglomeration trend of scenic spot distribution increased, changing into the aggregate spatial structure type. In 2009, the NNI of the Great Liupan Red Ecological Resort Plate was 0.71 with the aggregate-random distribution type of scenic spots, compared with the NNI of 0.44 in 2019. The trend of scenic spot aggregation distribution increased, and the spatial structure type changed from random type to aggregate type.

The spatial centroid mobility of scenic spots indicates the degree of change of the overall layout direction of tourist attractions in the region. The analysis of the change of the standard deviation ellipse area of the distribution of A-level rural tourist attractions in the seven tourism plates from 2009 to 2019 is shown in Figure 9. The elliptical direction of each tourism plate is consistent with the distribution of the whole province. Under the influence of the “The Belt and Road Initiative,” the number of plate attractions increases, but the centroid moves southwest.

Through the analysis of the spatial accessibility of rural tourist attractions in Ningxia, as shown in Figure 10, the time cost of scenic spot accessibility changed significantly at the provincial level from 2009 to 2019. The change rate of one-hour isochronous circle was 41.67%, the change rate of the isochronous circle of 1-2 hours was 1.95%, the change rate of the isochronous circle of 2-3 hours was 15.19%, and the change rate of three-hour isochronous circle was negative. Meanwhile, the spatial distribution of accessibility of scenic spots shows an increasing trend from the scenic spots along the main traffic arteries to the periphery. The areas with better accessibility are contiguously distributed around the traffic arteries and cities, while the rural scenic spots with poor accessibility are distributed in the rugged terrain of the provincial boundary.

## 5. Conclusion

The rural tourism attractions in Ningxia Hui Autonomous Region are selected as the research object to investigate the current situation of the spatial pattern of rural tourist attractions. Meanwhile, a spatiotemporal CNN model based on multifactor weighting is constructed to evaluate the spatial pattern of rural tourism. Through simulation, it is found that the constructed CNN model has high prediction accuracy of 97.69% and can effectively evaluate the spatial pattern, which can provide experimental basis for the digital development of rural tourism spatial pattern in the later stage.

## 6. Future Work

The evaluation and analysis of the spatial pattern of rural tourism reveal that although it can make a more accurate and effective evaluation, there are also some deficiencies. For example, in the spatial pattern analysis of scenic spot accessibility, only the impact of land transportation on rural tourism space in Ningxia is evaluated, and aviation is not included in the accessibility cost resistance model. In addition, the research only selects tourism destinations and transportation routes and lacks the relevant analysis of market factors.

In the future research direction, on the one hand, it is necessary to extend the research time limit, include market factors, explore the advantages and disadvantages of cluster development between plates, consider the impact of natural factors such as terrain and climate and human factors like social economy on accessibility, include aviation into the accessibility cost resistance model for evaluation, and minimize the calculation error of accessibility index value. On the other hand, in the future research, it is required to break the administrative boundaries and build a global tourism cooperation development model, to provide reference for the development of rural tourism economy and the improvement of spatial pattern.

## Figures and Tables

**Figure 1:** Diagram of the study area.

**Figure 2:** Requirements of rural tourism on the spatial pattern.

**Figure 3:** Process of feature extraction of rural tourism spatial pattern via the multifactor-weighted spatiotemporal CNN algorithm.

**Figure 4:** The comparison result of accuracy among the model and other deep learning algorithms.

**Figure 5:** The comparison result of precision among the model and other deep learning algorithms.

**Figure 6:** The comparison result of recall among the model and other deep learning algorithms.

**Figure 7:** The comparison result of *F*1 value among the model and other deep learning algorithms.

**Figure 8:** The comparison of NNI of the seven tourism plates in (a) 2009 and (b) 2019 (BK1: Great Sand Lake Holiday and Leisure Area; BK2: Xixia Cultural Tourism District; BK3: Saishang Hui Township Cultural Experience Plate; BK4: Frontier Cultural Tourism Plate; BK5: Great Shapotou Resort and Leisure Plate; BK6: Weizhou Historical and Cultural Tourism Plate; BK7: Great Liupan Red Ecological Resort Plate).

**Figure 9:** Change in the area of the standard deviation ellipse of A-level rural tourist attractions in the seven tourism plates in (a) 2009 and (b) 2019 (BK1: Great Sand Lake Holiday and Leisure Area; BK2: Xixia Cultural Tourism District; BK3: Saishang Hui Township Cultural Experience Plate; BK4: Frontier Cultural Tourism Plate; BK5: Great Shapotou Resort and Leisure Plate; BK6: Weizhou Historical and Cultural Tourism Plate; BK7: Great Liupan Red Ecological Resort Plate).

**Figure 10:** The change of time cost of spatial accessibility of rural tourist attractions in Ningxia in (a) 2009 and (b) 2019.

## Data Availability

The data used to support the findings of this study are available from the corresponding author upon request.
